The article "Emerging research trends in artificial intelligence for cancer diagnostic systems: A comprehensive review" was retracted in 2025. Reasons: unreliable results or conclusions; concerns about the citations.

# Emerging research trends in artificial intelligence for cancer diagnostic systems: A comprehensive review

**DOI:** 10.1016/j.heliyon.2024.e36743

**Published:** 2024-08-23

**Authors:** Sagheer Abbas, Muhammad Asif, Abdur Rehman, Meshal Alharbi, Muhammad Adnan Khan, Nouh Elmitwally

**Affiliations:** a Department of Computer Science, Prince Mohammad Bin Fahd University, Al-Khobar, KSA; b Department of Computer Science, Education University Lahore, Attock Campus, Pakistan; c School of Computer Science, National College of Business Administration and Economics, Lahore, 54000, Pakistan; d Department of Computer Science, College of Computer Engineering and Sciences, Prince Sattam Bin Abdulaziz University, 11942, Alkharj, Saudi Arabia; e Riphah School of Computing & Innovation, Faculty of Computing, Riphah International University, Lahore Campus, Lahore, 54000, Pakistan; f School of Computing, Skyline University College, University City Sharjah, 1797, Sharjah, United Arab Emirates; g Department of Software, Faculty of Artificial Intelligence and Software, Gachon University, Seongnam-si, 13120, Republic of Korea; h Department of Computer Science, Faculty of Computers and Artificial Intelligence, Cairo University, Giza, 12613, Egypt; i School of Computing and Digital Technology, Birmingham City University, Birmingham, B4 7XG, UK

**Keywords:** Machine learning deep learning, Artificial intelligence, Cancer diagnostics, Federated learning, Explainable AI

## Abstract

This review article offers a comprehensive analysis of current developments in the application of machine learning for cancer diagnostic systems. The effectiveness of machine learning approaches has become evident in improving the accuracy and speed of cancer detection, addressing the complexities of large and intricate medical datasets. This review aims to evaluate modern machine learning techniques employed in cancer diagnostics, covering various algorithms, including supervised and unsupervised learning, as well as deep learning and federated learning methodologies. Data acquisition and preprocessing methods for different types of data, such as imaging, genomics, and clinical records, are discussed. The paper also examines feature extraction and selection techniques specific to cancer diagnosis. Model training, evaluation metrics, and performance comparison methods are explored. Additionally, the review provides insights into the applications of machine learning in various cancer types and discusses challenges related to dataset limitations, model interpretability, multi-omics integration, and ethical considerations. The emerging field of explainable artificial intelligence (XAI) in cancer diagnosis is highlighted, emphasizing specific XAI techniques proposed to improve cancer diagnostics. These techniques include interactive visualization of model decisions and feature importance analysis tailored for enhanced clinical interpretation, aiming to enhance both diagnostic accuracy and transparency in medical decision-making. The paper concludes by outlining future directions, including personalized medicine, federated learning, deep learning advancements, and ethical considerations. This review aims to guide researchers, clinicians, and policymakers in the development of efficient and interpretable machine learning-based cancer diagnostic systems.

The article "Emerging research trends in artificial intelligence for cancer diagnostic systems: A comprehensive review" was retracted in 2025. Reasons: unreliable results or conclusions; concerns about the citations.

## 1 Introduction

Cancer diagnosis is a critical step in the effective treatment and management of cancer patients. Timely and accurate detection of cancer is vital for determining the appropriate treatment approach and improving patient outcomes. However, the increasing complexity and heterogeneity of cancer pose significant challenges to traditional diagnostic methods. In recent years, machine learning has become a pivotal tool in cancer diagnostics, providing opportunities to improve accuracy, efficiency, and personalized treatment decisions [[1], [2], [3]].

AI and machine learning (ML) are increasingly integrating into everyday life, especially within digital healthcare. These technologies are anticipated to greatly influence disease diagnosis and treatment soon. Advances in AI and ML have resulted in the creation of autonomous diagnostic tools that leverage large datasets to identify diseases in their early stages, with a particular emphasis on cancer detection. As a subset of AI, ML utilizes neural networks and algorithms that allow machines to learn and address problems in a manner akin to the human brain [4]. The objective of deep learning (DL), which is a subset of machine learning (ML), is to replicate the information processing methods of the human brain [5]. It is capable of image and object recognition, language processing, improving drug discovery, enhancing precision medicine, optimizing diagnostic procedures, and aiding human decision-making [6]. DL can also operate independently, suggesting outputs without human intervention [7]. Deep learning (DL) utilizes artificial neural networks (ANNs) designed to mirror the structure of the human brain, enabling the processing of various data types, including medical images. By integrating input, output, and numerous hidden layers, DL enhances the computational power of machine learning, enabling more sophisticated analysis and interpretation of complex datasets [8].

Deep Learning (DL) is revolutionizing various industries, such as healthcare, climate change [9], agriculture [10], and more. With DL, computers surpass trained human operators in tasks like picture categorization, object identification, and landmark location. The transformative potential of Machine Learning (ML) is widely recognized by experts, particularly in redefining the interpretation of imaging data. Although the medical imaging field is still in its early stages of utilizing these powerful technologies, it holds great promise. Medical imaging has the potential to facilitate personalized therapies tailored to individual needs and address the limited medical expertise available in developing nations [11].

The article "Emerging research trends in artificial intelligence for cancer diagnostic systems: A comprehensive review" was retracted in 2025. Reasons: unreliable results or conclusions; concerns about the citations.

Without explicit programming, computers can already identify patterns and anticipate outcomes from massive datasets thanks to machine learning techniques [12]. Machine learning algorithms may classify data, find hidden patterns, and create prediction models by utilizing statistical models and algorithms [[13], [14], [15], [16], [17], [18], [19], [20], [21]]. These capabilities make machine learning highly effective for analyzing complex medical data, such as imaging, genomics, and clinical records, and extracting meaningful insights for cancer diagnosis. The significance of machine learning in cancer diagnostics is highlighted by its ability to handle extensive and high-dimensional datasets. As technology rapidly advances, large amounts of data are generated in various formats, such as medical images, genomic sequences, and electronic health records. Machine learning algorithms can effectively process and analyze these data types, revealing critical insights that can aid in cancer detection and prediction [12,22,23].

This review article aims to deliver a comprehensive examination of the most recent trends in machine learning applications for cancer diagnostic systems as shown in Fig. 1. By investigating the current state-of-the-art machine learning methods, their applications, and the challenges they present, this review aspires to provide valuable insights and recommendations for researchers, clinicians, and policymakers involved in the development and implementation of effective and accurate cancer diagnostic systems. We will analyze various machine learning techniques utilized in cancer diagnosis, including supervised learning algorithms like Support Vector Machines (SVM), Random Forests (RF), and Neural Networks (NN) [[24], [25], [26]]. Furthermore, unsupervised learning algorithms, including clustering techniques, Principal Component Analysis (PCA), and Autoencoders, will be examined. The expanding domain of deep learning, featuring Convolutional Neural Networks (CNN), Recurrent Neural Networks (RNN), and Generative Adversarial Networks (GAN), will also be thoroughly discussed regarding their potential applications in cancer diagnosis [27]. Furthermore, we will delve into data acquisition and preprocessing methods specific to cancer diagnostics, encompassing imaging data such as biopsy and radiology images, genomic data including DNA sequencing and gene expression data, and clinical data derived from electronic health records and patient demographics [[28], [29], [30]]. The review will address feature extraction and selection techniques tailored to each data type, emphasizing image analysis, genomic mutation analysis, and clinical biomarker analysis.

The article "Emerging research trends in artificial intelligence for cancer diagnostic systems: A comprehensive review" was retracted in 2025. Reasons: unreliable results or conclusions; concerns about the citations.

**Fig. 1:** Flow diagram for systematic review conducted.

Model training and evaluation are crucial aspects of machine learning for cancer diagnosis, and this review will explore the methodologies employed in these processes. We will discuss the importance of training and validation datasets, evaluation metrics, and cross-validation techniques. This review will assess the performance of diverse machine learning models in the context of cancer diagnostics and will explore their applications across a range of cancer types, such as breast, lung, prostate, colorectal, and leukemia, among others. By examining the distinct challenges and opportunities presented by each cancer type, this article aims to illustrate how machine learning can significantly improve diagnosis, prognosis, and treatment strategies for individual patients.

Challenges and limitations associated with machine learning for cancer diagnosis will be addressed, including limited and imbalanced datasets, interpreting black-box models, integrating multi-omics data, and ethical and legal considerations. Furthermore, this article will delve into the emerging field of explainable artificial intelligence, which aims to make machine learning models more interpretable and transparent in healthcare settings. Additionally, future directions in the field will be outlined, such as personalized medicine and precision oncology, the integration of federated learning to address data privacy concerns, advancements in deep learning for cancer diagnosis, and the ethical considerations involved in deploying AI systems in clinical practice.

Explainable Artificial Intelligence (XAI) is critical in cancer diagnoses, increasing model transparency and certainty. Random Forests and decision trees aid in the identification of crucial predictive markers in breast cancer, hence enhancing diagnostic accuracy and interpretation [31]. SHAP values applied to deep learning models improve lung cancer diagnosis by revealing the influence of variables such as smoking history. LIME helps colorectal cancer patients by clarifying CNN judgments and highlighting crucial image regions for pathologists. Stanford University developed attention-based deep learning models for breast cancer mammography that improved accuracy, with visual explanations supporting radiologists. In prostate cancer, SVMs with feature attribution enhanced comprehension of recurrence factors, allowing for more customized care. CNNs with Grad-CAM for melanoma detection increased accuracy and trust by aligning model explanations with dermatologist thinking. These examples highlight XAI's involvement in improving diagnostics [32].

The article "Emerging research trends in artificial intelligence for cancer diagnostic systems: A comprehensive review" was retracted in 2025. Reasons: unreliable results or conclusions; concerns about the citations.

The paper begins with a brief introduction to artificial intelligence (AI), machine learning (ML), deep learning (DL), federated learning (FL), and explainable artificial intelligence (XAI). It underscores the current advancements in these fields and their practical applications in cancer research, as well as their potential future implications. This narrative literature review serves the following purposes.

• To enhance public understanding of AI, ML, DL, FL, and XAI and their significant contributions to cancer research. It aims to engage readers from diverse professions who may not be familiar with the technical intricacies of these technologies.
• To exclusively evaluate AI, ML, DL, FL, and XAI approaches. These techniques have demonstrated their suitability for image categorization, particularly in recent times. The focus of this work is primarily on utilizing deep learning techniques for image-based cancer diagnosis.
• To provide clear insights to readers regarding the most effective image modality for specific types of cancer diagnosis, including their advantages and disadvantages, as well as recent clinical trials conducted in this field.
• To verify and highlight the applicability of various pre-trained models for real-time cancer diagnosis across different types of cancer.
• To outline the expected accuracy of existing methods and propose potential improvements for the current techniques.

By pursuing these objectives, the paper seeks to share valuable knowledge and promote advancements in the application of AI, ML, DL, FL, and XAI in cancer research as shown in Fig. 2. In conclusion, this comprehensive review offers an in-depth analysis of the emerging trends in machine learning for cancer diagnostic systems. By exploring the current state-of-the-art approaches, applications, challenges, and future directions, the article aims to provide meaningful insights and guidance for developing and implementing efficient, accurate, and interpretable machine learning-based cancer diagnostic systems.

**Fig. 2:** Application of AI, ML, and DL in digital healthcare [36].

The article "Emerging research trends in artificial intelligence for cancer diagnostic systems: A comprehensive review" was retracted in 2025. Reasons: unreliable results or conclusions; concerns about the citations.

## 2 Artificial intelligence in cancer diagnosis

Artificial intelligence (AI) has become a valuable asset in cancer diagnosis, leading to numerous advancements and improvements as shown in Fig. 3. AI algorithms are capable of analyzing medical images, including mammograms, CT scans, and pathology slides, to detect early signs of cancer and assist in accurate diagnoses. These algorithms aid radiologists in identifying and classifying abnormalities, such as tumors or lesions, with exceptional precision and efficiency. A major advantage of AI in cancer diagnosis is its capacity to identify cancer in its early stages. By processing extensive patient data and medical records, AI algorithms can uncover subtle patterns and markers that may signal the presence of cancer, often before any visible symptoms arise.

**Fig. 3:** Artificial intelligence in cancer detection.

AI can provide decision support to healthcare professionals by offering recommendations based on vast amounts of patient data, research papers, and treatment guidelines. These systems can assist doctors in determining the most appropriate treatment plans for individual patients, taking into account factors such as tumor characteristics, genetic profiles, and treatment outcomes from similar cases. AI can contribute to personalized cancer care by analyzing patients' genomic data and predicting treatment responses. By considering genetic variations, AI algorithms can help identify targeted therapies that are likely to be more effective and reduce the risk of adverse reactions. This approach enables tailored treatment plans for individual patients, optimizing outcomes and reducing unnecessary treatments. AI can analyze clinical data to generate prognostic models, predicting patient outcomes and survival rates based on various factors such as age, tumor stage, biomarker expression, and treatment history. Additionally, AI algorithms can predict treatment response and identify potential relapse risks, aiding in treatment planning and follow-up care. AI algorithms have the ability to integrate and analyze extensive cancer-related data from various sources, such as electronic health records, research databases, and medical literature. This capability enables the identification of valuable insights, patterns, and associations that may not be easily recognizable to human researchers. By utilizing AI's data mining capabilities, scientists and clinicians can acquire new knowledge and enhance cancer diagnosis and treatment strategies. Additionally, AI can facilitate quality improvement in cancer diagnosis by offering consistency and standardization in the evaluation process. By automating certain tasks, such as image analysis or data extraction, AI reduces the potential for human error and variability, leading to more reliable and reproducible results [37,38].

The article "Emerging research trends in artificial intelligence for cancer diagnostic systems: A comprehensive review" was retracted in 2025. Reasons: unreliable results or conclusions; concerns about the citations.

**Table:** 

Authors	ML	DL	FL	Year	Methods	Results
Lorenzo et al. [39]	✓	×	×	1999	Multivariate Cluster Analysis	/
Kinkel [40]	×	✓	×	2002	CNN	Accuracy (83.11 %)
Markey et al. [41]	×	✓	×	2003	Invasive Exome Analysis	Accuracy (90 %)
Frangioini j [42]	×	✓	×	2008	CNN	Accuracy (93 %)
Fischerova et al. [43]	×	✓	×	2014	CNN	Accuracy (97 %)
Esteva et al. [44]	×	✓	×	2017	Inception v3 CNN	AUC (over 91 %)
Samala et al. [45]	×	✓	×	2018	DCNN	AUC (0.85 ± 0.05)
Coudary et al. [46]	×	✓	×	2018	DCNN	AUC (0.733–0.856)
Wu et al. [47]	✓	×	×	2018	Bayesian network	/
Yi a et al. [48]	✓	×	×	2018	Decision Tree J48	Accuracy (80 %)
Haenssle et al. [49]	×	✓	×	2018	Google's inception v4 CNN	Sensitivity (86.6%–88.9 %)
Chang et al. [50]	✓	×	×	2018	RTSE + CETRUS	Accuracy (86.2 %)
Li et al. [51]	×	✓	×	2019	DCNN	Sensitivity (93.4 %),
Zhu et al. [52]	×	✓	×	2019	CNN	Sensitivity (76.47 %)
Brancati et al. [53]	✓	×	×	2019	Convolutional Autoencoder, Supervised	F-measure Score Improved (5.06 %)
Tabibu et al. [54]	×	✓	×	2019	CNN	Accuracy (92.61 %)
Wang et al. [55]	×	✓	×	2019	CNN	Sensitivity 94.38 % Specificity 95.92 %
Zhang et al. [56]	×	✓	×	2019	Shear Wave Elastography	Sensitivity varies from 65 to 85 % Specificity varies from 33 to 82 %
Wu et al. [57]	×	✓	×	2019	CNN	Accuracy (90.4 %)
Han et al. [58]	×	✓	×	2019	Ultrasound + Shear Wave Elastography	Accuracy (80.4 %)
Gamage et al. [59]	×	✓	×	2019	CNN	Accuracy (66.07 %)
Poturnayova et al. [60]		✓	×	2019	CNN	Accuracy (97 %)
Duggento et al. [61]	×	✓	×	2019	CNN	Accuracy (98.3 %)
Vivarelli et al. [62]	×	✓	×	2019	CNN	Accuracy (78.5 %)
Ebigbo et al. [63]	×	✓	×	2020	CNN	Accuracy (89.9 %)
Poon et al. [64]	×	✓	×	2020	CNN	Polyp-based Sensitivity: 96.875 % Specificity: 92.9 %
Li et al. [65]	×	✓	×	2020	CNN	Sensitivity 98.04 % Specificity 95.03 %
Guo et al. [66]	×	✓	×	2020	CNN	Accuracy (98.7 %)
Hashimoto et al. [67]	×	✓	×	2020	CNN	Accuracy (95.414 %)
Aburaed et al. [68]	✓	×	×	2020	FFNN	Accuracy (99.3 %)
Hmoud et al. [69]	×	✓	×	2021	CNN	Accuracy (99.98 %)
Hohn et al. [70]	×	✓	×	2021	CNN	Accuracy (83 %)
Aggarwal et al. [71]	×	✓	×	2021	CNN	Accuracy (98.3 %)
Fu et al. [72]	×	✓	×	2021	CNN	Accuracy (99 %)
Zebai et al. [73]	×	×	✓	2021	Transfer Learning	Accuracy (99 %)
Sarma et al. [74]	×	×	✓	2021	Federated Learning	Accuracy (89.5 %)
Stephan et al. [75]	✓	×	×	2022	ANN	Specificity Level (90 %)
Dhier et al. [76]	✓		×	2022	FFNN	Accuracy (99.3 %)
Fati et al. [77]		✓	×	2022	CNN	Accuracy (83 %)
Ma z et al. [78]	×	×	✓	2022	Federated Learning	Accuracy (90 %)
Goudarzi et al. [79]	×	✓	×	2023	MRI/Ultrasound CNN + Augmented reality + optical 3D sensor	The error values of the three-dimensional views were 0.75, 0.99, and 0.80 respectively
Tan et al. [80]	×	×	✓	2023	Federated Learning	Accuracy (99.743 %)

While AI demonstrates significant potential in cancer diagnosis, it is essential to view it as a supportive tool rather than a substitute for healthcare professionals. The expertise and judgment of clinicians remain crucial in interpreting AI-generated insights and making informed decisions for patient care. Precision oncology, an innovative approach in the battle against cancer, revolves around the meticulous identification and characterization of individual tumor cells, and Artificial Intelligence (AI) plays a vital role in advancing this field [[81], [82], [83]]. By harnessing the power of AI, precision oncology targets specific molecular markers, offering a highly effective treatment strategy. This innovative approach is closely associated with personalized cancer genomic data and also utilizes proteomics data sourced from electronic health records maintained in various computational databases.

The article "Emerging research trends in artificial intelligence for cancer diagnostic systems: A comprehensive review" was retracted in 2025. Reasons: unreliable results or conclusions; concerns about the citations.

Recently, clinical oncology has experienced significant advancements due to the integration of AI-based molecular strategies. The use of next-generation sequencing (NGS) platforms has produced extensive high-throughput data, providing a foundation for further innovations. To leverage this data effectively, oncology experts with machine learning expertise are crucial. Their skills allow them to develop algorithms that promote early-stage cancer detection by identifying new biomarkers and target sites. Furthermore, these algorithms enhance diagnostic accuracy through NGS sequencing and the identification of specific target areas. Additionally, AI technology has greatly improved high-resolution medical imaging, leading to more precise and detailed cancer diagnoses [[84], [85], [86]].

Precision oncology drugs are specifically designed to target cancer cells based on their unique genetic profiles. By leveraging NGS data, AI algorithms can recommend effective therapies that consider personalized genetic factors. As a result, AI is regarded as one of the most promising approaches for precise cancer diagnosis, prognosis, and treatment. The systematic analysis of data from pharmaceutical and clinical big datasets empowers AI to provide comprehensive insights. Consequently, the future of healthcare and clinical practices is anticipated to shift toward algorithm-driven AI support for tasks such as radiology image analysis, electronic health record management, and data mining. This shift will facilitate the delivery of more accurate and tailored solutions for cancer treatment [[87], [88], [89]].

The article "Emerging research trends in artificial intelligence for cancer diagnostic systems: A comprehensive review" was retracted in 2025. Reasons: unreliable results or conclusions; concerns about the citations.

## 3 Machine learning in cancer diagnosis

Cancer is a complex and devastating disease that continues to pose a significant global health challenge. The World Health Organization (WHO) reports that cancer is among the leading causes of death worldwide, accounting for millions of fatalities annually. Early and accurate diagnosis is vital for enhancing patient outcomes and increasing survival rates. However, diagnosing cancer presents a considerable challenge, often necessitating extensive medical expertise, time-consuming analyses of medical images and laboratory tests, and a thorough understanding of intricate molecular signatures [[33], [34], [35], [36], [90], [91]].

Oncology has seen a revolution in the use of machine learning (ML) techniques for cancer diagnosis in recent years. Within the field of artificial intelligence, machine learning (ML) offers computational techniques that let computers learn from data and make judgments or predictions without requiring explicit programming. Through the use of large-scale datasets and sophisticated algorithms, machine learning models have proven to be exceptionally adept at identifying important patterns and insights from complex medical data, including genetic information, radiological images, and clinical notes [[92], [93], [94]]. This research paper seeks to examine the substantial influence of machine learning on cancer diagnosis and its potential to revolutionize healthcare practices in the direction of precision medicine. By leveraging the capabilities of ML, researchers and clinicians can improve the accuracy, efficiency, and speed of cancer diagnosis, resulting in more personalized and targeted treatment strategies.

The integration of ML in cancer diagnosis offers several key advantages. Firstly, it enables the development of predictive models that can identify high-risk individuals who are prone to developing certain types of cancer. This facilitates early intervention and the implementation of preventive measures, potentially reducing cancer-related morbidity and mortality rates. Additionally, ML algorithms can aid in the classification and differentiation of various cancer subtypes, enabling tailored treatment plans and personalized therapies [95,96]. Additionally, ML techniques can enhance the analysis of medical imaging data, including computed tomography (CT), magnetic resonance imaging (MRI), and positron emission tomography (PET) scans. These powerful algorithms can accurately detect and characterize tumor lesions, assess their growth patterns, and predict their response to specific treatments. Such advancements are particularly crucial in optimizing treatment decisions, minimizing unnecessary procedures, and reducing patient burden.

The article "Emerging research trends in artificial intelligence for cancer diagnostic systems: A comprehensive review" was retracted in 2025. Reasons: unreliable results or conclusions; concerns about the citations.

Furthermore, the integration of ML with genomic profiling has unlocked new avenues for precision medicine in cancer diagnosis [97]. By analyzing vast genomic datasets, ML algorithms can identify genetic alterations, biomarkers, and gene expression patterns associated with specific cancers. This information can be utilized to create robust predictive models for prognosis, treatment response, and drug resistance, assisting clinicians in making informed decisions about patient management. However, challenges remain in the adoption and implementation of machine learning in cancer diagnosis. These challenges include issues related to data quality and availability, ethical considerations, the interpretability of machine learning models, and regulatory concerns. Overcoming these obstacles necessitates interdisciplinary collaboration among clinicians, data scientists, and policymakers to ensure the responsible and effective use of machine learning-based diagnostic tools.

In conclusion, there is a great deal of promise for precision medicine in healthcare practices through the use of machine learning techniques in cancer detection. Machine learning has the potential to improve the precision, efficacy, and personalized aspect of cancer diagnosis by utilizing sophisticated algorithms and vast quantities of medical data. The future of cancer care is expected to be shaped by the integration of machine learning in oncology, which will ultimately improve patient outcomes and dramatically lower the cancer burden worldwide as long as researchers and doctors keep coming up with new ideas and solutions to these problems.

Since its founding in 1956, artificial intelligence (AI) has advanced significantly with the aim of building machines that can replicate human thought processes and reasoning in challenging jobs. Machine learning (ML) is a prominent area of artificial intelligence that has grown in popularity. ML uses algorithms to evaluate data, find patterns, and produce insightful information that can be used to make decisions. Within the larger subject of AI, machine learning (ML) has become a potent tool in the context of cancer diagnosis. The virtues and disadvantages of machine learning and deep learning (DL) as separate approaches are highlighted in Fig. 2, which depicts significant turning points in AI research. These methodologies have distinct features and are applicable in multiple fields. Scientists have demonstrated that these methods have the potential to improve diagnostic capacities by adapting and applying them in the field of cancer precision medicine. The purpose of this review is to examine the various AI techniques, their subtleties, and examples of how clinical specialists apply them to cancer analysis [98,99].

The article "Emerging research trends in artificial intelligence for cancer diagnostic systems: A comprehensive review" was retracted in 2025. Reasons: unreliable results or conclusions; concerns about the citations.

Furthermore, as Fig. 2 illustrates, AI research has expanded into a number of sub-disciplines, including expert systems, fuzzy logic, computer vision, natural language processing, and recommendation systems. This has increased the field's influence on clinical research. At its core, machine learning (ML) employs algorithms to analyze data, reveal hidden patterns, and generate insights, facilitating predictions and informed decision-making in real-world applications. In contrast to traditional software programs designed for specific tasks, ML algorithms undergo a training process using extensive datasets to dynamically learn and accomplish various tasks. DL, on the other hand, represents a subset of ML, relying on deep neural networks trained through supervised or unsupervised learning modes.

The exponential growth of DL has introduced novel learning techniques, such as the residual network, positioning DL as a distinct learning method. However, it is essential to recognize that ML serves as the realization of AI, while DL serves as a means to implement ML. Despite its progress, DL does exhibit limitations. Firstly, DL models necessitate substantial training data to achieve accurate results, which may be challenging in scenarios where biomedical samples are scarce. Secondly, in certain domains, traditional and simpler ML techniques prove sufficient for problem-solving, rendering complex DL methods unnecessary [[100], [101], [102]].

## 4 Deep learning in cancer diagnosis

As one of the main causes of death worldwide, cancer continues to have a significant negative impact on people's lives, families, and healthcare systems. Treatment planning, prognosis, and patient survival are significantly impacted by early detection and precise diagnosis. Conventional diagnostic techniques frequently rely on intrusive procedures and visual examination of tissue samples, which can cause delays in diagnosis and subpar results.

Deep learning methods have become extremely useful in a number of domains recently, such as speech recognition, computer vision, and natural language processing. Artificial neural networks, which are modelled after the composition and operation of the human brain, are used in deep learning to automatically extract hierarchical representations from large, complicated datasets [103,104]. This ability to extract intricate patterns and features from massive amounts of data has the potential to transform the area of cancer diagnosis [105,106]. With the application of deep learning techniques, the fields of radiology and pathology related to medical imaging have advanced significantly. Tumor features and behavior can be extensively inferred from medical imaging data, such as computed tomography (CT), magnetic resonance imaging (MRI), and histopathological slides. Using this data, deep learning algorithms can estimate patient outcomes, identify cancers, and extract important traits [107,108].

The article "Emerging research trends in artificial intelligence for cancer diagnostic systems: A comprehensive review" was retracted in 2025. Reasons: unreliable results or conclusions; concerns about the citations.

This research paper's primary objective is to present a comprehensive analysis of the most current developments in deep learning methods for cancer diagnosis. The several imaging modalities and techniques used, such as lung imaging, histopathology slides, and mammography, will be discussed in this article. Additionally, it will examine various deep learning architectures, highlighting the unique advantages and disadvantages of each, including generative adversarial networks (GANs), recurrent neural networks (RNNs), and convolutional neural networks (CNNs) [109,110]. Furthermore, the article will discuss the challenges and limitations associated with deep learning in cancer diagnosis. Issues such as dataset scarcity, interpretability, generalizability, and clinical adoption will be addressed. While deep learning has shown remarkable results in several studies, there are still obstacles that need to be overcome before its widespread implementation in clinical practice.

By highlighting the advancements and challenges in deep learning for cancer diagnosis, this research paper aims to offer researchers, clinicians, and policymakers’ valuable insights into the potential of this technology to transform cancer care. Ultimately, leveraging deep learning in cancer diagnosis could facilitate earlier detection, enhance prognostic accuracy, and enable personalized treatment strategies, significantly improving patient outcomes in the battle against cancer [111,112].

## 5 Federated learning in cancer diagnosis

Cancer diagnosis is a vital component in the detection and treatment of malignant tumors. However, the analysis of large volumes of medical data for accurate and timely diagnosis poses significant challenges, such as privacy concerns and restrictions on data sharing. To address these issues, the concept of federated learning has emerged as a promising solution within the healthcare sector. This research paper investigates the advancements and challenges related to the application of federated learning techniques in cancer diagnosis as shown in Fig. 4. By utilizing distributed datasets from multiple institutions while maintaining data privacy, federated learning has the potential to improve the accuracy and efficiency of cancer diagnostic models [113,114].

**Fig. 4:** Federated learning applications in healthcare.

The article "Emerging research trends in artificial intelligence for cancer diagnostic systems: A comprehensive review" was retracted in 2025. Reasons: unreliable results or conclusions; concerns about the citations.

Federated learning greatly improves cancer diagnostics by safeguarding patient privacy, facilitating collaborative data sharing, and enhancing model performance. In this approach, hospitals and research institutions can collaboratively train machine learning models using decentralized data sources while keeping raw patient data secure. For instance, multiple hospitals can collaborate on refining a lung cancer detection model by securely aggregating insights from locally stored imaging and clinical data. This ensures patient confidentiality while leveraging diverse datasets to enhance the model's accuracy and robustness. By aggregating local updates into a global model, federated learning facilitates the development of more effective diagnostic tools that can generalize well across different patient populations and healthcare settings, thereby advancing precision medicine in oncology [115].

Conventionally, medical data analysis necessitates gathering data into a single area, raising issues with data security, privacy, and HIPAA compliance. An option is offered by federated learning, which permits cooperative model training across decentralized data sources while maintaining data confidentiality and privacy. Federated learning principles in the context of cancer diagnosis entail a process that involves model aggregation, participant selection, and privacy-preserving methods including differential privacy and safe multi-party computation. With this technique, academics and healthcare organizations can work together to train models on local datasets without sharing sensitive patient data [116].

Recent advancements in federated learning have demonstrated significant potential in cancer diagnosis research. Numerous studies and projects have effectively utilized federated learning techniques to enhance diagnostic accuracy, improve predictive models, and optimize treatment plans. Integrating federated learning with emerging technologies such as artificial intelligence, deep learning, and computer vision further enhances the precision and personalization of cancer diagnostics [74]. Despite its potential benefits, federated learning in cancer diagnosis also faces challenges and limitations. Issues such as data heterogeneity, communication overhead, model convergence, bias and fairness, and regulatory compliance need to be addressed. Ethical implications and potential risks related to the implementation of federated learning models in healthcare must be thoughtfully addressed.

Looking ahead, future research directions for federated learning in cancer diagnosis include exploring federated transfer learning, meta-learning, and adaptive privacy mechanisms [117]. These advancements have the potential to enhance the effectiveness and efficiency of cancer diagnostic models. Federated learning offers a transformative approach that tackles data privacy concerns while advancing cancer diagnosis and improving patient care. By examining the advancements and challenges of federated learning in cancer diagnosis, this research paper provides valuable insights for researchers, healthcare practitioners, and policymakers interested in leveraging this innovative approach to enhance cancer detection and treatment.

The article "Emerging research trends in artificial intelligence for cancer diagnostic systems: A comprehensive review" was retracted in 2025. Reasons: unreliable results or conclusions; concerns about the citations.

## 6 Limitations and future direction

To tackle the challenge of interpretability in machine learning models used for cancer diagnostics, a promising future direction is the integration of Explainable Artificial Intelligence (XAI) techniques, such as fairness in prediction and explainability. XAI focuses on delivering human-understandable explanations for the decisions made by AI systems, allowing users to understand and trust the rationale behind the model's predictions as shown in Fig. 5. Research efforts should not only focus on traditional machine learning models but also explore the potential of federated learning techniques, as only a few studies have investigated their application in this domain. By using federated learning, where models are trained across multiple decentralized datasets without sharing raw data, it becomes possible to improve prediction accuracy while maintaining data privacy and security.

**Fig. 5:** Explainable AI model.

Moreover, the integration of XAI methods in combination with federated learning into existing machine learning frameworks designed for cancer diagnostics holds significant potential. These approaches can provide not only improved prediction accuracy but also transparent insights into the decision-making process. Techniques such as rule-based models, feature importance analysis, visualization tools, and model-agnostic explanations can be applied to federated learning models, enabling healthcare professionals to interpret the distributed knowledge learned from multiple sources.

Furthermore, the incorporation of federated learning and XAI techniques can enhance patient understanding and trust in the diagnostic process. Patients can receive comprehensible explanations about the factors influencing their diagnosis, even when their data is part of a larger, decentralized model. This aspect is crucial in healthcare, where patient privacy and trust are of utmost importance. By leveraging federated learning, healthcare institutions can collaborate and collectively improve diagnostic models without compromising patient data privacy.

The article "Emerging research trends in artificial intelligence for cancer diagnostic systems: A comprehensive review" was retracted in 2025. Reasons: unreliable results or conclusions; concerns about the citations.

In addition to the technical aspects, future research should also focus on the ethical implications and regulatory considerations associated with federated learning and XAI in cancer diagnostics. Developing guidelines that address data privacy, patient consent, and algorithmic fairness in the federated setting would further ensure the responsible deployment of these technologies in real-world clinical applications.

In conclusion, there is a lot of promise for overcoming interpretability issues, improving prediction accuracy, and fostering patient and healthcare professional trust by combining federated learning and XAI approaches into machine learning models for cancer diagnosis. Adopting these novel strategies and conducting additional research in this domain would allow the AI-driven healthcare sector to make significant progress toward more efficient, transparent, and private diagnostic solutions.

## 7 Conclusion

With its high levels of accuracy and predictive power, machine learning has emerged as a major asset for cancer detection systems. The inability of current machine learning models to be interpreted, however, is a significant drawback that erodes patient and healthcare provider acceptability and confidence. These models are "black-box," meaning that the logic underlying their predictions is hidden, making validation, error analysis, and further improvements more difficult.

A promising future path to address this restriction is the incorporation of Explainable Artificial Intelligence (XAI) techniques into machine learning frameworks for cancer diagnoses. XAI approaches aim to provide comprehensible and transparent justifications for the choices made by AI systems so that medical practitioners may comprehend and have faith in the logic underlying the model's forecasts. The interpretability gap can be closed by using XAI, which enables cooperation, validation, and the discovery of biases in AI systems and human experts. Additionally, integrating XAI techniques in cancer diagnostic systems enhances patient understanding and trust. Patients can receive comprehensible explanations about the factors influencing their diagnosis, empowering them to actively participate in their healthcare decisions. This patient-centered approach fosters a collaborative environment where patients are more informed and engaged in their treatment journey.

Future studies, however, should concentrate on the ethical issues and legal frameworks that surround the application of XAI techniques in addition to the development and improvement of these techniques. In AI-driven healthcare, uniform norms and best practices are necessary to guarantee accountability, openness, and adherence to moral principles. In conclusion, XAI approaches have the potential to close the interpretability gap and foster patient and healthcare professional trust in machine learning models for cancer diagnosis. This development will result in AI-driven healthcare solutions that are more morally sound, accountable, and transparent, which will eventually improve patient outcomes and diagnostic accuracy in the fight against cancer.

The article "Emerging research trends in artificial intelligence for cancer diagnostic systems: A comprehensive review" was retracted in 2025. Reasons: unreliable results or conclusions; concerns about the citations.

## Data availability

The authors confirm that the data supporting the findings of this study are available within the article.

## CRediT authorship contribution statement

**Sagheer Abbas:** Methodology, Data curation, Conceptualization. **Muhammad Asif:** Investigation, Formal analysis, Conceptualization. **Abdur Rehman:** Resources, Project administration, Investigation, Data curation. **Meshal Alharbi:** Writing – original draft, Resources, Project administration. **Muhammad Adnan Khan:** Validation, Supervision, Software, Resources. **Nouh Elmitwally:** Writing – original draft, Supervision, Methodology.

## Declaration of competing interest

The authors declare that they have no known competing financial interests or personal relationships that could have appeared to influence the work reported in this article.

Authors have not recieved any funding for this manuscript.
